The article "A Role for PPARγ in the Regulation of Cytokines in Immune Cells and Cancer" was retracted in 2015. Reasons: plagiarized text; duplicated text; overlap with other authors' work; overlap with earlier publications.

# A Role for PPAR*γ* in the Regulation of Cytokines in Immune Cells and Cancer

**DOI:** 10.1155/2008/961753

**Published:** 2008-06-12

**Authors:** Xiao Yi Yang, Li Hua Wang, William L. Farrar

**Affiliations:** ^1^Basic Research Program, SAIC-Frederick, National Cancer Institute-Frederick, Frederick, MD 21702, USA; ^2^Cancer Stem Cell Section, Laboratory of Cancer Prevention, Division of Basic Sciences, National Cancer Institute-Frederick, Frederick, MD 21702, USA

## Abstract

Peroxisome proliferator-activated receptor *γ* (PPAR*γ*) is a ligand-activated transcription factor and a member of the nuclear receptor superfamily. PPAR*γ* and its ligands appear to serve diverse biological functions. In addition to the well-studied effects of PPAR*γ* on metabolism and cellular differentiation, abundant evidence suggests that PPAR*γ* is an important regulator of the immune system and cancers. Since cytokines are not only key modulators of inflammation with pro- and anti-inflammatory functions but they also can either stimulate or inhibit tumor growth and progression, this review summarizes the role for PPAR*γ* in the regulation of cytokine production and cytokine-mediated signal transduction pathways in immune cells and cancer.

## 1. INTRODUCTION

Peroxisome proliferator-activated receptors (PPARs) are members of the nuclear receptor superfamily [1–6]. PPARs exist in three isoforms, PPAR*α*, PPAR*β*/*δ*, and PPAR*γ*, which are encoded by different genes and harbour isotype-specific expression patterns and functions. PPARs were initially identified as mediators of peroxisome proliferation in rodent liver, where PPAR*α* plays the major role. However, none of the PPARs could be attributed to peroxisome proliferation in humans [7–10]. Among the various subtypes of PPARs, PPAR*γ* is the best characterized receptor in humans. There are at least two PPAR*γ* isoforms derived from the alternative promoters, PPAR*γ*1 and PPAR*γ*2. PPAR*γ*2 isoform is longer than PPAR*γ*1 by additional 30 N-terminal amino acids [11, 12]. Synthetic ligands including the thiazolidinedione (TZD) class of drugs, L-tyrosine-based compounds, and diindolymethanes as well as natural ligands including a broad range of polyunsaturated fatty acids 9- and 13-hydroxyoctadecadienoic acid (9- and 13-HODE) and the eicosanoids 15-deoxy-Δ^12, 14^-prostaglandin J2 (15-d-PGJ2) function as efficacious PPAR*γ* activators [13–15].

PPAR*γ* is expressed at high levels in adipose tissue and is an important regulator of adipocyte differentiation, which functions as a ligand-dependent, sequence-specific activator of transcription. Expression of PPAR*γ* in immune system was initially documented in 1994. Kliewer et al. reported that PPAR*γ* is expressed at high levels in mouse spleen [8]. Greene et al. detected the expression of PPAR*γ*2 in normal neutrophils and peripheral blood lymphocytes by Northern blot analysis in 1995 [9]. Monocytes and macrophages were the first cells of the immune system in which the physical presence and anti-inflammatory properties of PPARs were first described [16, 17]. Subsequently, PPAR*γ* has been reported to exist in other immune cell types of hematopoietic origin, including T lymphocytes [18–22], B lymphocytes [23], NK cells [24], dendritic cells [25–28], eosinophils [29], and mast cells [30–32].

The article "A Role for PPARγ in the Regulation of Cytokines in Immune Cells and Cancer" was retracted in 2015. Reasons: plagiarized text; duplicated text; overlap with other authors' work; overlap with earlier publications.

Multiple lines of evidence suggest that PPARs, especially PPAR*γ*, are known to be expressed or overexpressed in several cancers such as epithelial tumor cells, renal cell carcinoma cells, myeloid and lymphoid malignancies, and multiple myeloma cells [33–37]. Ligands of PPAR*γ* have been shown to promote differentiation and to inhibit cell growth and induce apoptosis in several types of human cancer, including colon cancer [38–40], breast cancer [41, 42], lung cancer [43], prostate cancer [44, 45], gastric cancer [46], liposarcoma [47, 48], and leukaemia [49], supporting a role for PPAR*γ* ligands as potential tumor suppressors in PPAR*γ*-dependent or -independent manner [50, 51], although several murine models suggest that, under certain circumstances, PPAR*γ* ligands may stimulate cancer formation [36].

The cytokines are a large family of secreted molecules consisting of more than 100 peptides or glycoproteins. Each cytokine is secreted by particular cell types in response to a variety of stimuli and produces a characteristic constellation of effects on the growth, motility, differentiation, or function of its target cells. Cytokines can act in an autocrine manner to affect the behavior of the cell that releases the cytokine and/or in a paracrine manner to affect the behavior of adjacent cells. Moreover, some cytokines are stable enough to act in an endocrine manner to affect the behavior of distant cells, although this depends on their abilities to enter the circulation and their half-life in the blood. Cytokines are especially important for regulating immune and inflammatory responses with pro- and anti-inflammatory functions, and have crucial functions in controlling both the innate and adaptive arms of the immune response. Not only do cytokines govern the development and homeostasis of lymphocytes, but they also direct the differentiation of helper T cells and promote the generation of memory cells [52]. During formation and development of tumor, the mixture of cytokines that is produced in the tumor microenvironment has an important role in cancer pathogenesis. Cytokines can either stimulate or inhibit tumor growth and progression [53–57]. Specific polymorphisms in cytokine genes are associated with an increased risk of cancer [58]. Cytokines are produced by immune cells as a host response to cellular stress caused by either exogenous or endogenous agents to control and minimize cellular damage. However, an uncontrolled and sustained generation of cytokines can lead to altered cell growth, differentiation, and apoptosis. Therefore, cytokines are a linker among immunity, inflammation, and cancer [59].

The article "A Role for PPARγ in the Regulation of Cytokines in Immune Cells and Cancer" was retracted in 2015. Reasons: plagiarized text; duplicated text; overlap with other authors' work; overlap with earlier publications.

In addition to their antiproliferative and proapoptotic activities on immune cells and cancer cells, effects of PPARs and their ligands in immune system and cancer cells may be mediated through influencing cytokine production or cytokine-mediated signal transduction pathways. Conversely, the expression of PPARs is also modulated by cytokines. In this review, we recapitulate molecular mechanisms on PPARs regulating cytokine production or cytokine-mediated signal transduction and cell responses, and enumerate their physiological and pathological consequences in immune responses, inflammation, and cytokine-responsive tumors.

## 2. MECHANISM(S) OF CYTOKINE GENE REGULATION BY PPAR*γ*

Like other nuclear receptors, the structure of PPARs is comprised of: an amino-terminal activation function, AF-1 (A/B domain), which can activate transcription in a ligand-independent fashion, the DNA-binding domain (DBD), a hinge region, and a carboxy-terminal ligand-binding domain (LBD) [1–3, 60, 61]. The DBD allows them to bind to and activate target genes, thus defining them as transcription factors. The LBD also contains a second activation function (AF-2) that maps to a surface-exposed hydrophobic pocket, proving a docking site for coregulatory proteins, and modulates their activities, making them hormone-dependent transcription factors. Upon ligand binding, PPARs heterodimerize with retinoid X receptors (RXRs) and form a complex that translocates to the nucleus and regulates gene expression. This heterodimeric complex binds to peroxisome proliferator response elements (PPREs) located within the promoter regions of target genes that consist of a direct repetition of the consensus AGGTCA half-site spaced by one or two nucleotides (DR1 or DR2). In addition to the heterodimer complex, it has been reported that a host of accessory proteins, named “coactivators” or “corepressors,” bind to the nuclear receptors PPAR/RXR in a ligand-dependent manner and impact the transcriptional process by either remodeling chromatin structure and/or acting as adapter molecules that link the nuclear receptor complex to key transcriptional machinery. Ligand binding to PPARs appears to trigger conformational changes that permit their dissociation from corepressors and favor their association with coactivators. The coactivators possess or recruit histone acetyltransferase activity to the transcription site. Subsequently, acetylation of histone proteins alters chromatin structure, thereby facilitating the binding of RNA polymerase and the initiation of transcription. In the absence of ligand, PPAR*γ* has the potential to silence genes to which it is bound by recruiting transcriptional corepressor complexes and repress gene expression [1–5, 62, 63, 64].

The article "A Role for PPARγ in the Regulation of Cytokines in Immune Cells and Cancer" was retracted in 2015. Reasons: plagiarized text; duplicated text; overlap with other authors' work; overlap with earlier publications.

Surprisingly, most of the effects of PPARs on cytokine expression result from crosstalk with other transcriptional factors through nongenomic transrepressive mechanisms. It is well known that some key transcriptional factors such as nuclear factor of activated T cells (NFAT), nuclear factor-kappa B (NF-*κ*B), GATA-3, T-bet, AP-1, or signal transducers and activators of transcription (STAT) regulate the expression of cytokine genes. Transrepression by PPARs can occur either by inhibiting the binding of transcriptional factors to DNA through direct protein to protein interactions or by sequestrating cofactors necessary to their activity. A protein-to-protein interaction between PPARs and other transcription factors completely prevents these transcription factors from binding to their own response elements and therefore blocks their transcriptional activation of cytokine genes [63, 64]. Activation of PPAR*γ* negatively influences the production of inflammatory cytokines such as tumor necrosis factor-alpha (TNF*α*), Interleukin (IL)-6, and IL-1*β* by macrophages. A well-established example is PPAR*γ* coassociation with NFAT, a T-cell specific transcription factor, in regulation of IL-2 gene expression [18]. The transcription factor NFAT plays an essential role in gene expression of IL-2 by T lymphocytes and is also involved in the proliferation of peripheral T lymphocytes. Therefore, we evaluated transcriptional activity and DNA binding of NFAT to determine whether NFAT might be a target for negative regulation of T-cell activation by PPAR*γ* ligands. Utilizing the gel-shift experiment, we found that PPAR*γ* ligands significantly inhibited the specific binding of NFAT probe corresponding to the human IL-2 promoter. The transcriptional activation of the reporter construct directed by the NFAT distal site of the IL-2 promoter was abrogated by 15-d-PGJ_2_ or ciglitazone in the presence of PPAR*γ* over expression. We further tested for complex formation between PPAR*γ* and NFAT in a coimmunoprecipitation experiment. The NFAT can be coprecipitated with PPAR*γ* in T cells induced by PMA/PHA and 15-d-PGJ_2_ or ciglitazone. Furthermore, the addition of anti-PPAR*γ* antibody induced high-affinity binding of extracts to the NFAT probes as determined by using an electronic mobility shift assay, demonstrating that removal of PPAR*γ* with this antiserum increases the target specificity of NFAT. This data indicated that a direct physical protein-protein interaction occurs between nuclear receptor PPAR*γ* and transcription factors NFAT, in turn inhibiting transcription of IL-2 in T lymphocytes.

The article "A Role for PPARγ in the Regulation of Cytokines in Immune Cells and Cancer" was retracted in 2015. Reasons: plagiarized text; duplicated text; overlap with other authors' work; overlap with earlier publications.

## 3. CROSSTALK OF PPAR*γ* WITH CYTOKINE-MEDIATED SIGNAL TRANSDUCTION PATHWAYS

 Cytokines induce a variety of biological responses by binding to specific cell surface receptors and activating cytoplasmic signal transduction pathways, such as the Janus kinase-signal transducer and activator of transcription (JAK-STAT) pathway, which transmits information received from extracellular polypeptide signals, through transmembrane receptors, directly to target gene promoters in the nucleus, providing a mechanism for transcriptional regulation without second messengers [65–74]. JAKs bind specifically to intracellular domains of cytokine receptor signaling chains and catalyze ligand-induced phosphorylation of themselves and of intracellular tyrosine residues on the receptor, creating STAT docking sites. Phosphorylation of STATs on activating tyrosine residues leads to STAT homo- and heterodimerization. STAT dimers are rapidly transported from the cytoplasm to the nucleus and are competent for DNA binding. Binding of the activated STAT dimer to a target promoter initials formation of a primary transcription complex and dramatically increases the transcription rate from this promoter of target gene. Transcription of target genes induced by the STAT dimers reflects an intrinsic ability of STAT transcriptional activation domains to recruit nuclear coactivators that mediate chromatin modifications and communication with the core promoters [73].

Several lines of evidence indicated that activated PPAR*γ* crosstalks with cytokine-mediated signal transduction pathways in modulation of immune responses and tumor cell growth and apoptosis [75–82]. Interestingly, in the case of interactions between PPAR*γ* and STAT3 [83–87], two structurally distinct PPAR*γ* ligands suppress IL-6 activated-STAT3 through the divergent types of crosstalk including direct or a corepressor SMRT-mediated association (see Figure 1). The 15-d-PGJ2 is a naturally occurring ligand with low affinity of PPAR*γ*, whereas a class of antidiabetic drugs known as thiazolidinediones is a type of high-affinity synthetic ligands of PPAR*γ*. Because the ligand-binding pocket is not static, each PPAR*γ* ligand has the potential to induce a different conformation of the receptor. Additionally, a non-PPAR*γ*-dependent mechanism may be involved in the difference between the effects of 15-d-PGJ2 and the thiazolidinediones on STAT3. Therefore, it is reasonable that these two structurally distinct PPAR*γ* agonists suppress IL-6 activated STAT3 through diverse molecular mechanisms. The multiplicity of crosstalk between nuclear receptors and other transcriptional factors is an important factor that contributes to both signal diversification and specification.

 Direct protein-protein interaction between transcription factors and ligand-activated nuclear receptors has been shown involved in the regulation of some transcription factors. In multiple myeloma cells, we demonstrated that upon 15-d-PGJ2 binding, PPAR*γ* indeed interacted with phosphorylated STAT3 and represses IL-6 signaling by inhibiting the binding of STAT3 to target genes [84]. Ligand-induced activation of PPAR*γ* induces growth arrest by antagonizing the prosurvival signaling cascade induced by IL-6. PPAR*γ* impedes IL-6 signaling by inhibiting the transcription of a number of STAT3-regulated genes such as mcl-1 and c-myc that are important in cell growth and survival. The exact mechanism through which PPAR*γ* represses STAT3 has not been fully elucidated. PPAR*γ* has been shown to physically associate with STAT3, which may inhibit STAT3 from binding DNA or possibly facilitate the export of STAT3 out of the nucleus. However, certain agonists that induced growth arrests of these cells did not induce SMRT to dissociate from PPAR*γ*, suggesting that this nuclear hormone receptor may use numerous mechanisms to inhibit multiple myeloma cell growth.

The article "A Role for PPARγ in the Regulation of Cytokines in Immune Cells and Cancer" was retracted in 2015. Reasons: plagiarized text; duplicated text; overlap with other authors' work; overlap with earlier publications.

An alternative mechanism for PPAR*γ*-mediated STAT3 repression has also been suggested, in which PPAR*γ* agonist treatment of multiple myeloma cells induces the corepressor protein SMRT to dissociate from PPAR*γ*; SMRT could then complex with and inhibit the transcriptional activities of STAT3. The corepressor SMRT has also to be demonstrated to mediate PPAR*γ* downregulation of STAT3 in multiple myeloma cells. PPAR*γ* can form weak interactions with the corepressor NCoR/SMRT complex. PPAR*γ* cannot bind to DNA while it is associated with the corepressor complex. After ligand binding, PPAR*γ* disassociates from the corepressor complex, and then binds to DNA through a peroxisome proliferator response element. We first clarified that treatment of MM cells with troglitazone decreased association of SMRT with PPAR*γ*, which results in redistribution of corepressor SMRT from PPAR*γ* to activated STAT3. Furthermore, this interaction between SMRT and IL-6-activated STAT3 can be attenuated by a PPAR*γ* antagonist GW9662, confirming the specificity of the exchange of corepressor SMRT induced by the liganded PPAR*γ*. Recruitment of SMRT, which is associated with histone deacetylase, by STAT3 leads to transcriptionally inactivating STAT3 and consequently downregulating IL-6 mediated MM cell growth and gene expression. These observations support that coactivators or corepressors function is not only for regulation of the ligand-dependent DNA binding and transcriptional activities of nuclear receptors themselves but also acts as a bridge protein to modulate nuclear receptors crosstalk with other transcription factors.

The article "A Role for PPARγ in the Regulation of Cytokines in Immune Cells and Cancer" was retracted in 2015. Reasons: plagiarized text; duplicated text; overlap with other authors' work; overlap with earlier publications.

## 4. PPAR REGULATION OF CYTOKINE IN IMMUNE CELLS

The immune response can be classified into two fundamental types: innate and adaptive immunity. The innate immune response functions as the first line of defense against infection. It consists of soluble factors, such as complement proteins, and diverse cellular components including granulocytes (basophils, eosinophils, and neutrophils), mast cells, macrophages, dendritic cells, and natural killer cells. The adaptive immune response is slower to develop but manifests as increased antigenic specificity and memory. It consists of antibodies, B cells, and CD4^+^ and CD8^+^ T lymphocytes. Natural killer T cells and *γ* *δ*T cells are cytotoxic lymphocytes that straddle the interface of innate and adaptive immunity [57]. In immune responses innate and adaptive immunity are interlocked and complement each other.

Signaling in the immune system can be either a direct interaction of cells or be mediated by cytokines and antibodies that are carrying signals to all cells with the appropriate receptors. Although PPAR*γ* involvement in the regulation of innate immunere sponses has been studied since the late 1990s [16, 17], only recently it has the role of PPAR*γ* in adaptive immunity been investigated [18–32]. Here, we focus on PPAR*γ* regulation of cytokine-mediated immune responses in immune cells.

### 4.1. PPAR and IL-2

IL-2 is an autocrine and paracrine growth factor that is secreted by activated T lymphocytes and is essential for clonal T cell proliferation. Although originally described as a potent T cell growth factor in vitro, the main nonredundant role of IL-2 in vivo is now known to be the maintenance of peripheral T cell tolerance. As well as promoting the proliferation and survival of recently activated effector T cells, IL-2 also plays a critical role in regulatory T cell (Treg) homeostasis and has been variously described as promoting the thymic development, peripheral homeostasis and suppressive function of Tregs. These observations, stemming largely from studies on various murine models of IL-2 and IL-2 receptor deficiency, have prompted a greater understanding of the protolerogenic nature of IL-2 dependent signaling.

The article "A Role for PPARγ in the Regulation of Cytokines in Immune Cells and Cancer" was retracted in 2015. Reasons: plagiarized text; duplicated text; overlap with other authors' work; overlap with earlier publications.

Greene et al. detected the expression of PPAR*γ*2 in normal neutrophils and peripheral blood lymphocytes in 1995 [9]. In human peripheral blood T cells, we detected inhibition of PHA-induced proliferation and IL-2 production by 15-d-PGJ_2_ and TZD troglitazone in a dose-dependent manner [18]. When PPAR*γ*2 wild type expression vector was transfected into Jurkat cells, we found that troglitazone and 15-d-PGJ_2_ inhibited transcription and production of IL-2 in Jurkat cells in a PPAR*γ*-dependent manner. Cotransfection assays with PPAR*γ* and PPRE-driven/IL-2 promoter luciferase reporter constructs revealed that the inhibitory effects of troglitazone and 15-d-PGJ_2_ on IL-2 promoter activity are dependent on the expression and activation of PPAR*γ*. Finally, we demonstrated that activated PPAR*γ* inhibited the DNA-binding and activity of transcription factor NFAT regulating the IL-2 promoter in T cells.

Clark et al. described the expression and function of PPAR*γ* in mouse T-lymphocytes [20]. They demonstrated that murine SJL-derived Th1 clones and freshly isolated T cell-enriched splenocytes from SJL mice express PPAR*γ*1 mRNA but not PPAR*γ*2. To test its functional significance, they used two PPAR*γ* ligands, 15-d-PGJ_2_ and a TZD, ciglitazone. Both ligands could inhibit antigen-induced and anti-CD3 antibody-induced T cell proliferative responses of T cell clones, and the freshly isolated T cell enriched splenocytes. In these studies, it was also demonstrated that the two PPAR*γ* ligands mediated inhibition of IL-2 secretion by the T cell clones, whereas inhibition of IL-2 induced proliferation was not detected.

### 4.2. PPAR and IL-4

IL-4 is a pleiotropic and multifunctional cytokine produced by activated T cells, mast cells, and basophils [88]. IL-4 plays a critical role in regulating the outcome of an immunere sponse by facilitating the differentiation of CD4^+^ T cells into IL-4-producing T helper (Th) type 2 cells and suppressing the differentiation of interferon-*γ* producing Th1 cells, thereby favoring humoral immune responses [89]. Regulation of IL-4 gene expression, therefore, is critically important for the differentiation of Th2 cells and Th2-dependent immune responses [90]. Dysregulated expression of IL-4-producing cells has been linked with autoimmune and allergic diseases [91].

In T cells, IL-4 gene expression is regulated at the transcriptional level by both ubiquitous and cell type-restricted factors, including NF-AT, c-Maf, GATA-3, STAT6, JunB, and other transcription factors [90]. These factors interact with a proximal promoter region composed of multiple regulatory elements that can both positively and negatively affect transcriptional activation. IL-4 gene transcription is mediated by subset-specific transcription factors such as GATA-3 and c-Maf during the differentiation of naive T cells into Th2 cells. A phase of short-term gene transcription, elicited by the interaction of differentiated T cells with antigen, requires the antigen-induced transcription factor NFAT. Treatment of CD4^+^ T cells with ciglitazone or 15-d-PGJ2 triggered the physical association between PPAR*γ* and NFATc1, resulting in IL-4 promoter inhibition and decreased IL-4 production [92].

The article "A Role for PPARγ in the Regulation of Cytokines in Immune Cells and Cancer" was retracted in 2015. Reasons: plagiarized text; duplicated text; overlap with other authors' work; overlap with earlier publications.

Huang et al. [93] reported that IL-4 induces expression of PPAR*γ* and 12/15-lipoxygenase in macrophages, suggesting the potential of coordinated induction of both receptor and activating ligands. Therefore, it appears likely that PPAR*γ* is a key factor in regulating at least some aspects of macrophage lipid metabolism and primarily as a repressor of inflammatory responses. The ways how these two processes are connected, and the contribution of macrophage specific PPAR*γ*-induced gene expression and transrepression to inflammatory responses in vivo remains to be explored.

We reported an interesting PPAR*γ* ligand-mediated immunoregulatory circuit between monocyte/macrophages and T cells [19]. Traditionally, T helper cells can be divided into two functional subsets consisting of Th1 and Th2 cells on the basis of the immunoregulatory cytokines that these T cells produce. Some of these immunoregulatory cytokines possess cross-regulatory properties and can enhance or suppress cytokine production by Th1 or Th2 subset. Thp cells are the pluripotent precursors of Th1 and Th2 cells. Moreover, the development of either Th1 or Th2 helper cells is believed to be determined by the effects of cytokines directly on helper Thp cells. IL-4 is principally produced by helper T cells of theTh2 phenotype. IL-4 has been shown to induce 12/15 lipoxygenase in monocytes/macrophages, which converts arachidonic acid into several metabolic products, including the potential PPAR*γ* ligand 13-HODE [93]. Based on this finding, we tested the relevance of the regulation of soluble mediators (PPAR*γ* ligands) released by IL-4 treated monocytes/macrophages on T cell activation. The medium of macrophages cultured with or without IL-4 was added to T cells stimulated with anti-CD3 or PHA/PMA. We found that T cells with the conditioned medium from IL-4-treated macrophages produced significantly less IL-2. The medium of IL-4-treated macrophages contained a sufficient amount of 13-HODE and anti-13-HODE antibody could neutralize the inhibitory effects of the IL-4-conditional medium on T cell IL-2 production. Using human T lymphocytes and the PPAR*γ*-transfected Jurkat T cells, we demonstrated the specific inhibition by 13-HODE of the transcription factors NFAT and NF-*κ*B, the IL-2 promoter reporter, and IL-2 production. These observations led us to hypothesize that IL-4, produced by Th2 cells, may indirectly affect the production of IL-2 by Thp or Th1 helper cells by inducing the production of these potential PPAR*γ* ligands by macrophage 12/15-lipoxygenase, which in turn interferes with the subsequent development of T helper cells (see Figure 2) [19].

The article "A Role for PPARγ in the Regulation of Cytokines in Immune Cells and Cancer" was retracted in 2015. Reasons: plagiarized text; duplicated text; overlap with other authors' work; overlap with earlier publications.

Since many complicated pathological situations cannot be simply explained by the Th1 cell and Th2 cell paradigm, efforts to resolve these issues in recent years have resulted in the discovery of many new T helper cell subsets such as Treg cell and Th17 cell subsets. Therefore, it is interesting to explore further how PPAR*γ* regulates these new Th subsets (see Section 5).

### 4.3. PPAR and IFN*γ*

IFN*γ* plays a central role in inflammatory reactions and is predominately produced by CD4, CD8, and NK cells. IFN*γ* drives inflammatory reactions by stimulating the release of NO, TNF-*α*, and IL-1*β* bymonocytes/macrophages. IFN*γ* is also a major effector cytokine, responsible for driving cell-mediated immunity and mediating organ-specific autoimmunity. Recent studies have shown that PPAR*γ* ligands inhibit IFN*γ* production by T lymphocytes; however, the mechanism underlying this observation has not been clarified [94]. Based on previous studies, PPAR*γ* ligands could indirectly decrease IFN*γ* by inhibiting activation of T cells, production of IL-2, or induction of apoptosis, or inhibiting IL-12 production by antigen-presenting cells [95–98].

 Cunard et al. demonstrated that PPAR*γ* is expressed in both murine CD4 and CD8 cells and that PPAR*γ* ligands directly decrease IFN*γ* expression by murine and transformed T cell lines. In contrast, GW9662, a PPAR*γ* antagonist, increases IFN*γ* expression. Transient transfection studies reveal that PPAR*γ* ligands, in a PPAR*γ*-dependent manner, potently repress an IFN*γ* promoter construct. Repression localizes to the distal conserved sequence of the minimal IFN*γ* promoter. They also demonstrate that PPAR*γ* acts on the minimal IFN*γ* promoter by interfering with c-Jun activation. These studies suggest that many of the observed anti-inflammatory effects of PPAR*γ* ligands may be related to direct inhibition of IFN*γ* by PPAR*γ* [94].

## 5. PPAR REGULATION OF CYTOKINES IN TH17 AND REGULATORY T CELLS

Recently, Th17 cells and CD4^+^ CD25^+^ regulatory T (Treg) cells have been described as two distinct T helper cell subsets from Th1 and Th2 cells. Th17 cells play critical roles in the development of autoimmunity and allergic reactions by producing IL-17 and, to a lesser extent, TNF-*α* and IL-6 [99, 100], while Treg cells expressing the forkhead/winged helix transcription factor (Foxp3) have an anti-inflammatory role and maintain tolerance to self components by contact-dependent suppression or releasing anti-inflammatory cytokines [transforming growth factor (TGF)-*β*1 and IL-10], therefore, the balance between Th17 and Treg may be important in the development/prevention of inflammatory and autoimmune diseases [101, 102].

The article "A Role for PPARγ in the Regulation of Cytokines in Immune Cells and Cancer" was retracted in 2015. Reasons: plagiarized text; duplicated text; overlap with other authors' work; overlap with earlier publications.

### 5.1. PPAR, IL-17 and Th17 cells

Production of IL-17 is a defining feature of a recently identified class of effector T cells termed Th17 cells [99, 100]. Th17 cells act as a distinct effector subset and secrete the signature cytokine IL-17, a proinflammatory cytokine that recruits and activates neutrophils, enhances T cell priming, and promotes the release of inflammatory mediators. Th17 cells provide defense against extracellular bacteria, mediate inflammation, and are critical for many types of autoinflammatory disorders (i.e., experimental autoimmune encephalomyelitis, type II collagen-induced arthritis, inflammatory bowel disease, and psoriasis). The discovery and initial characterization of these Th17 cells have provided a potential explanation for various chronic disease pathologies that were unclear with an understanding of only the Th1 and Th2 cell subsets.

IL-10-deficient (IL-10^−/−^) mice spontaneously develop inflammatory bowel disease with a Th1-polarized cytokine pattern. In addition to showing high colonic expression of the Th1-derived cytokine IFN*γ*, IL-10^−/−^ mice also show high expression of IL-17. Lytle et al. observed that rosiglitazone, a high-affinity ligand for PPAR*γ*, had its greatest effect in suppressing IL-17 production in IL-10 knockout mice [103]. Interestingly, the PPAR*α* ligand fenofibrate has been shown to repress IL-17 expression in cultured splenocytes activated by PMA plus ionomycin and by Th17 cells in a pathogenic CD4^+^ T cell line cultured from C3H Bir mice treated with cecal bacterial antigens [104].

### 5.2. PPAR, TGF*β* and Treg cells

At least two subtypes of CD4^+^ CD25^+^ regulatory T cells (Tregs) have been described: thymically derived natural Tregs (nTregs) and inducible Tregs (iTregs) generated peripherally from CD4^+^ CD25^−^ T effector cells (Teff) [100, 101]. Induced Treg are more functionally and phenotypically heterogeneous in comparison to natural Treg and can be subdivided into: induced Foxp3^+^ Tregs, Th3, and Tr1. Which signals drive Treg cell proliferation in the tumor setting? TGF*β* is the cytokine that is thought to foster Treg-cell amplification [101]. Both tumor cells directly or “tumor educated” immune cells can locally produce large amounts of TGF*β* [102]. Some mouse and rat tumors actively induce myeloid immature dentritic cells to secrete TGF*β* and this promotes Treg cell proliferation. There is also substantial evidence that indicates the involvement of TGF*β* in Treg cell conversion. Wohlfert et al. have used ciglitazone, a synthetic PPAR*γ* ligands, to characterize the relationship between PPAR*γ* ligands and both iTregs and nTregs. They reported that ciglitazone-activated PPAR*γ* enhances the TGF*β*-dependent conversion of naive T cells into Foxp3^+^-induced Tregs in vitro, although the mechanism by which PPAR*γ* enhances Treg activity remains unknown [105]. Hontecillas and Bassaganya-Riera have used PPAR*γ* deficient CD4^+^ cells obtained from tissue-specific PPAR*γ* null mice to investigate the role of endogenous PPAR*γ* on Treg and effector CD4^+^ T cell function. They demonstrated that only PPAR*γ*-expressing Treg was able to completely prevent inflammation induced by effector cells of either genotype, suggesting that PPAR*γ* expression and/or activation by endogenous agonists is required for optimal Treg function [106].

The article "A Role for PPARγ in the Regulation of Cytokines in Immune Cells and Cancer" was retracted in 2015. Reasons: plagiarized text; duplicated text; overlap with other authors' work; overlap with earlier publications.

## 6. PPAR REGULATION OF CYTOKINES IN CANCER CELLS

Cytokines that are released in response to infection, inflammation, and immunity can function to inhibit tumor development and progression. Alternatively, cancer cells can respond to host-derived cytokines that promote growth, attenuate apotosis, and facilitate invasion and metastasis. Proinflammatory cytokines implicated in carcinogenesis include IL-1, IL-6, IL-15, colony stimulating factors, TNF-*α*, and the macrophage migration inhibitory factor. A unique immune response signature, consisting predominantly of humoral cytokines, promotes metastasis in hepatocellular carcinoma. Likewise, a signature consisting of 11 cytokine genes in the lung environment predicted lymph node metastasis and prognosis of lung adenocarcinoma with *IL-8* and *TNF-*α** as the top 2 genes for predicting prognosis. *IL-8* was originally described as a monocyte-derived neutrophil chemotactic factor that specifically attracted neutrophils and was renamed due to its multiple function. *IL-8* can have angiogenic activities in several cancers including nonsmall cell lung cancer and can function as a positive autocrine growth factor. Both *TNF-*α** and *IL-6* contributed to the chemically induced skin tumors and lymphomas in mice. Collectively, cytokines are considered as a linker between inflammation and cancer [55–57].

The article "A Role for PPARγ in the Regulation of Cytokines in Immune Cells and Cancer" was retracted in 2015. Reasons: plagiarized text; duplicated text; overlap with other authors' work; overlap with earlier publications.

A considerable amount of research has shown that PPAR*γ* ligands suppress the proliferation rates of many types of cancer cells, particularly those derived from liposarcoma, colon cancer, breast cancer, prostate cancer, myeloid leukemia, glioblastoma, and many others. Various in vitro studies have shown that treatment of many types of cancer cells with TZD resulted in the induction of cell differentiation or apoptosis as well as improvement in levels of various markers for invasion and metastasis. Furthermore, activation of PPAR*γ* by glitazones inhibits angiogenesis and neovascularization both in vitro and in vivo and blocks the release of vascular endothelial growth factor from smooth muscle cells [107, 108]. In addition to the above direct antiproliferative and proapoptotic activities on cancer cells, effects of PPARs and their ligands in cancer cells may function through influencing cytokine production or cytokine-mediated signal transduction pathways. The mechanisms are probably linked to: (1) PPAR ligands may sensitize cancer cells to the antitumor effects of cytokines such as TNF*α*, (2) PPAR ligands may suppress production of cytokines for tumor cell growth, and (3) PPAR ligands may affect tumor microenvironment by regulation of Treg through influencing associated cytokines. A good example is that PPAR*γ* ligands suppress multiple myeloma through inhibiting IL-6 and IL-6 activated signal pathway in both PPAR*γ*-dependent and -independent manner.

### 6.1. PPAR and IL-6

Interleukin-6 (IL-6) is a cytokine with multiple biologic activities on a variety of cells. IL-6 plays a major role in the response to injury or infection and is involved in the immune response, inflammation, and hematopoiesis. Its deregulation impacts numerous disease states, including many types of cancer. Consequently, modulating IL-6 may be an innovative therapeutic strategy in several diseases. IL-6 is a pleiotropic cytokine that is involved in the physiology of virtually every organ system. Aberrant expression of this cytokine has been implicated in diverse human illnesses, most notably inflammatory and autoimmune disorders, coronary artery and neurologic disease, gestational problems, and neoplasms. In cancer, high levels of circulating IL-6 are observed in almost every type of tumor studied and predict a poor outcome. Furthermore, elevated IL-6 levels are associated strongly with several of the striking phenotypic features of cancer. Several molecules have been developed recently that target the biologic function of IL-6. Early results in the clinic suggest that this strategy may have a significant salutary impact on diverse tumors. The field of cytokine research has yielded a deep understanding of the fundamental role of IL-6 and its receptor in health and disease. Therapeutic targeting of IL-6 and its receptor in cancer has strong biologic rationale, and there is preliminary evidence suggesting that targeting of the IL-6 system may be beneficial in the treatment of cancer [109].

The article "A Role for PPARγ in the Regulation of Cytokines in Immune Cells and Cancer" was retracted in 2015. Reasons: plagiarized text; duplicated text; overlap with other authors' work; overlap with earlier publications.

One of the most studied tumor types in relation to IL-6 is multiple myeloma, a malignancy of differentiated B-lymphocytes. Multiple myeloma is characterized by accumulation of clonal plasma cells in the bone marrow, accounts for 10% of all hematologic cancers, and remains an incurable hematological malignancy [110–112]. Recently, we investigated how PPAR*γ* ligands suppress IL-6 gene expression through crosstalk between PPAR*γ* and NF-*κ*B or between PPAR*γ* and C/EBP*β* [86]. C/EBP*β* and NF-*κ*B bind to the promoter region of the IL-6 gene, and their cooperation is needed to activate IL-6 transcription. The nuclear receptor PPAR*γ* can be activated by troglitazone. Predominately, the complex between C/EBP*β* and troglitazone-bound PPAR*γ* leads to decreased DNA binding and transactivation of C/EBP*β*, inhibiting gene expression of IL-6. In addition, PGC-1, a coactivator, is shared by both PPAR*γ* and NF-*κ*B. After activation by ligands, ligand-bound PPAR*γ* competes for the limited amounts of PGC-1. Therefore, NF-*κ*B dissociates with PGC-1 and decreases NF-*κ*B DNA-binding and transactivation, leading to blocked IL-6 transcription. In the case of 15-d-PGJ2 inhibition of IL-6 transcription, although 15-d-PGJ2 also shares the above ligand-bound PPAR*γ* downregulation mechanisms on C/EBP*β* and NF-*κ*B, 15-d-PGJ2, compared with troglitazone, prefers to use PGC-1 as a bridging protein to associate with NF-*κ*B. In addition, 15-d-PGJ2 inactivates NF-*κ*B through decreasing phosphorylation of IKK and I*κ*B in PPAR*γ*-independent manner. The molecular mechanisms of PPAR*γ* ligands on the regulation of multiple transcription factors have proven, not surprisingly, complex. Given that IL-6 is the key growth and survival factor of multiple myeloma cells, and is particularly involved in the origin of all benign and malignant plasma cell expansions as well as MM cell resistance, the effects and targets of the PPAR*γ* ligands on aspects of multiple myeloma biology and bone marrow stromal cells may be clinically relevant.

## 7. CONCLUSIONS

Most proinflammatory cytokines produced by either host immune cells or tumor cells themselves promote tumor development. By contrast, proapoptotic and anti-inflammatory cytokines usually interfere with tumor development [55]. There is emerging evidence that the nuclear receptor PPAR*γ* interacts with transcriptional factors to modulate cytokine production and action in immunity, inflammation, autoimmune diseases, and tumors. PPAR*γ* regulation may occur at the levels of gene expression of cytokines themselves and their receptors or cytokine-mediated signaling transduction pathways in immune cells and cancer. The crosstalk between PPARs and cytokine signaling pathways mediating inflammatory effects at the cellular level is also effective to induce the expression of PPAR genes. The molecular basis of this interaction has remained elusive, despite the proposal of several distinct mechanisms. One of the most important mechanistic aspects is protein-protein interaction through a direct or cofactor-mediated indirect manner. On the basis of insights into the mechanisms on interaction between these two distinct families of transcriptional factors activated by different signaling pathways, new targeting drug design and/or therapeutic strategies will be discovered and developed for treatment of cytokine-related diseases ranging from inflammation to cancer.

The article "A Role for PPARγ in the Regulation of Cytokines in Immune Cells and Cancer" was retracted in 2015. Reasons: plagiarized text; duplicated text; overlap with other authors' work; overlap with earlier publications.

## Figures and Tables

**Figure 1:** *PPAR*γ* crosstalk with IL-6-activated STAT3 signaling pathway.* Upon IL-6 binding, the IL-6R/gp130 dimer induces phosphorylation of JAK1,3, which in turn phosphorylates STAT3. The phosphorylated STAT3 dimerizes and translocates to the nucleues, where they bind to the STAT3 binding element (SBE) in the responsive gene to initiate transcription. Two structurally distinct PPAR*γ* agonists suppress IL-6-activated STAT3 through diverse molecular mechanisms. 15-d-PGJ2 enhances direct physical protein-protein interaction between PPAR*γ* and phosphorylated STAT3 and represses IL-6 signaling by inhibiting the binding of STAT3 to target promoters; Troglitazone inhibits the interaction between PPAR*γ* and the corepressor SMRT, thereby inducing the redistribution of SMRT from PPAR*γ* to activated STAT3, in turn transcriptionally inactivating STAT3 signaling.

**Figure 2:** *PPAR*γ* regulation of cytokine-mediated immunoregulatory circuit between monocytes/macrophages and T lymphocytes.* T helper (Th) lymphocytes can be traditionally divided into two functional subsets consisting of Th1 and Th2 cells on the basis of the immunoregulatory cytokines that these T cells produce. Thp cells are the pluripotent precursors of Th1 and Th2 cells. IL-4 is principally produced by helper T cells of theTh2 phenotype. IL-4 can induce the upregulation of expression of the enzyme 12/15 lipoxygenase in monocytes/macrophages, providing a potential PPAR*γ*-specific ligands 13-HODE. The mediator secreted by monocytes can be taken up by neighboring Thp or Th1 cells and activate PPAR*γ* in these cells. Since NFAT and NF-*κ*B bind to the promoter region of the IL-2 gene and are needed to activate IL-2 transcription in T cells, the ligand-dependent binding of PPAR*γ* to NFAT and NF-*κ*B correlates the dissociation of NFAT and NF-*κ*B from IL-2 promoter, thus inhibiting gene expression of IL-2 in Thp or Th1 cells.

The article "A Role for PPARγ in the Regulation of Cytokines in Immune Cells and Cancer" was retracted in 2015. Reasons: plagiarized text; duplicated text; overlap with other authors' work; overlap with earlier publications.

## ABBREVIATIONS

AF: Activation function
AP-1: Activation protein 1
C/EBP: CCAT/enhancer-binding protein
DBD: DNA binding domain
ER: Estrogen receptor
IFN: Interferon
IL: Interleukin
Jaks: Janus kinases
LBD: Ligand binding domain
MAPK: Mitogen-activated protein kinase
MM: Multiple myeloma
NcoR: Nuclear receptor corepressor
NFAT: Nuclear factor of activated T cells
NF-*κ*B: Nuclear factor-kappa B
PPAR: Peroxisome proliferator-activated receptor
PPRE: PPAR response element
RAR: Retinoic acid receptor
RXR: Retinoid-X receptor
STAT: Signal transducer and activator of transcription
SMRT: Silencing mediator of retinoid and thyroid receptors
SRC: Steroid receptor coactivator
TGF: Transforming growth factor
Th: T helper cell
TNF: Tumor necrosis factor
Treg: Regulatory T cell
TZD: Thiazolidinedione.
